# microRNA-16 Via Twist1 Inhibits EMT Induced by PM2.5 Exposure in Human Hepatocellular Carcinoma

**DOI:** 10.1515/med-2019-0078

**Published:** 2019-09-15

**Authors:** Hao Zhang, Zhihu Li

**Affiliations:** 1 School of Civil Engineering and Architecture, Anhui University of Technology, Ma’anshan, Anhui 243032, China

**Keywords:** microRNA-16, Human hepatocellular carcinoma, PM2.5

## Abstract

Epidemiological study has confirmed that PM2.5 (particulate matter with an aerodynamic diameter less than 2.5 μm) is associated with the incidence and progression of human hepatocellular carcinoma (HCC). Accordingly, this study was undertaken to investigate the pro-metastatic effects of PM2.5 on human HCC cell line SMMC-7721 in vitro and to explore the underlying mechanisms. CCK-8 assay was performed to examine the effect of PM2.5 on the proliferation of SMMC-7721 cells; scratch wound assay and transwell matrigel system has been used to examine the effect of PM2.5 on the migration and invasion ability of SMMC-7721 cells; furthermore, effect of PM2.5 on epithelial mesenchymal transition (EMT) of SMMC-7721 cells were examined by examining the EMT markers vimentin, ɑ-smooth muscle actin (ɑ-SMA), and E-cadherin; furthermore, the roles of microRNA-16 (miR-16) and its target Twist1 in PM2.5 induced carcinogenic effects were also examined. Results of CCK-8 assay suggested that PM2.5 promoted the proliferation of SMMC-7721 cells in a dose and time dependent manner. PM2.5 also markedly promoted the migration and invasion ability of SMMC-7721 cells. Moreover, epithelial mesenchymal transition (EMT) was also triggered by PM2.5. On the other hand, microRNA-16 (miR-16) and its target Twist1 was found to be mediated by PM2.5, and miR-16 mimic could suppress the metastatic ability of SMMC-7721 cells exposure to PM2.5 via inversely regulating the expression of Twist1. Furthermore, dual Luciferase reporter assay confirmed the specifically binding of miR-16 to the predicted 3′-UTR of Twist1. The present study confirmed the pro-proliferative and pro-metastatic effect of PM2.5 on HCC cell line SMMC-7721. The possible mechanisms were EMT process induced by PM2.5 in SMMC-7721 cells, which was accompanied by a decrease in miR-16 and increase in Twist1 expression.

## 1 Introduction

Air pollution has gradually become one of the major environmental issues in China and causes human health problems [1, 2]. Particulate matter (PM) refers to microscopic solid or liquid particles suspended in air, which is the major factors affecting air quality [3, 4]. PM2.5 (PM with an aerodynamic diameter less than 2.5 μm) is generally used to assess the severity of air pollution [5, 6]. PM2.5 mainly originates from human daily activities such as fuel combustion, and its surface is enriched with a large number of inorganic and organic components. The chemical composition of the PM2.5 include sulfate, nitrate, ammonium salt, metal oxides and minerals, which is very different due to the different sources of pollution [7, 8].

PM has been listed as a human carcinogen by International Agency for Research on Cancer [9, 10]. Associations between high PM2.5 concentration and lung cancer development have been well-investigated [11, 12]; however, the associations between PM 2.5 and other cancers have received less attention. PM2.5 may also target the liver which can induce oxidative stress, inflammation and genotoxicity [13, 14, 15], and a recent study provided suggestive evidence that ambient PM2.5 could increase the risk of liver cancer, accelerating liver steatosis and liver cancer progression [16, 17]. For example, people exposure to PM2.5 showed increased serum levels of hepatic enzymes such as alanine aminotransferase, a key marker of liver damage and a predictor of the most common liver cancer hepatocellular carcinoma (HCC) [18, 19]. It has been reported that PM2.5 was able to induce metastasis in HCC cell lines SMMC-7721 and HuH-7 [20], and tumor metastasis is acknowledged as the major cause of HCC development [19].

Epithelial mesenchymal transition (EMT) is a cellular trans-differentiation program that enables polarized, immotile epithelial cells to convert to motile mesenchymal cells. There is growing evidence that EMT contributes to tumor migration and invasion, indicating the hallmarks of malignancy [21]. Activation of EMT is characterized by loss of adhesion, up-regulation of the mesenchymal markers such as vimentin and ɑ-SMA, and down-regulation of the epithelial markers such as E-cadherin.

miRNAs are a group of small non-coding RNAs (18-22 nucleotides), which are involved in various cellular functions (including EMT) by regulating the expression of the target mRNAs through binding to their 3’- UTR [22, 23]. miR-16 has been reported to be abnormally expressed in HCC and the enhancement of miR-16 could repress the proliferation, invasion, and metastasis of HCC cells by mediating EMT process [24]. Twist1, an important EMT transcription factor known to suppress E-cadherin transcription, is identified as the direct target of miR-16. Twist1 has been suggested to have oncogenic properties and the expressions of miR-16 and Twist1 in cancer cells and tissues were inversely correlated [25, 26]. Evidence shows that Twist1 regulates the expression of several EMT-related genes to mediate tumor cells [27, 28, 29].

Here we confirmed the pro-proliferative and pro-metastatic effect of PM2.5 on HCC cell line SMMC-7721, analyzed the potential of PM2.5 on EMT transition in SMMC-7721 cells, and then investigated whether miR-16-1-3p and its target Twist1 was involved in PM2.5 induced metastasis and EMT transition.

## 2 Methods and materials

### 2.1 Cell culture and PM2.5 treatment

Human hepatocellular carcinoma cell line SMMC-7721 was obtained from Shanghai Biological Cell Bank (Shanghai, China). Cells were cultured in RPMI-1640 medium (Gibco, USA) supplemented with 10% fetal bovine serum and 1% antibiotic-antimycotic agent (Thermo Fisher Scientific Inc, USA). Cells were incubated in a humidified atmosphere at 37°C containing 5% CO2 and passaged at 80% confluence using 0.25% trypsin. Cells in logarithmic growth phase were cultured in a concentration gradient of PM2.5 solution (0, 5, 25, 50 μg/ml) for different time. PM2.5 was purchased from Sigma-Aldrich, Inc. (St. Louis, MO, USA). The control group received the same volume of incomplete RPMI-1640 medium.

### 2.2 Transfection

SMMC-7721 cells were transfected with miR-16-1-3p mimic or negative control using Lipofectamine 2000 reagent (Invitrogen, Carlsbad, USA) following the manufacturer’s protocol. The miR-16-1-3p and the negative control was provided by RiboBio (Guangzhou, China). Transfection efficiency was determined at 48h post-transfection using real-time quantitative PCR (RT-qPCR). Transfected cells were then used for further experiments.

### 2.3 Proliferation assay

SMMC-7721 cells were seeded at a density of 5×10^3^ cells/ well in a 96-well culture plate. Triplicate samples of growing cells were treated with a concentration gradient of PM2.5 solution as indicated above for different time (0, 12, 24, 48h). Medium was then replaced with a fresh PM2.5-free medium and cell proliferation was assessed with Cell Counting Kit-8 (CCK-8) assay (Promega, USA). Following the manufacturer’s protocol, 10 μl of CCK-8 solution was added to each well and the cells were subsequently incubated for 2h at 37°C. The optical density was then measured at 450 nm and the results were expressed as a percentage of control.

### 2.4 Western blotting

SMMC-7721 cells or the transfected cells were treated in 25 μg/ml of PM2.5 solution for 48h. After treatments, cells were washed with ice-cold PBS and lysed with 500 μl lysis buffer containing a protease inhibitor cocktail (Roche, Basel, Switzerland) on ice for 30 min with vortex every 5 min. Cell debris was removed by centrifugation at 12000 x g for 10 min at 4°C, and the protein concentration was determined with Bio-Rad protein assay kit (Bio-Rad, USA). Cell lysate was boiled for 5 min in 1 × SDS loading buffer. An equal amount of protein (50 μg) was then resolved on a 10 % sodium dodecylsulfate polyacrylamide gels (SDS– PAGE) and then transferred to polyvinylidene difluoride (PVDF) membranes. The membranes were blocked in 5% skim milk in phosphate buffer solution (PBS) containing 0.5% Tween for 2 h at room temperature, then incubated at 4 °C with the appropriate concentration of various antibodies. After hybridization with primary antibodies, the membranes were washed with PBS for five times, then incubated with Horseradish Peroxidase (HRP)-conjugated secondary antibodies (dilution, firm) for 30 min at room temperature and washed with PBS five times. Final detection was performed using ECL reagent (Millipore, USA) and imaged with a Bio-Rad imaging system. The intensity of target bands was quantified using Quantity One software with GAPDH as a loading control. The antibodies were as follows: anti-α-SMA (dilution, firm), anti-E-cad-herin (dilution, firm), anti-Vimentin (dilution, firm), and anti-Twist1 (dilution, firm) antibody.

### 2.5 RT-qPCR

SMMC-7721 cells or the transfected cells were treated in 25 μg/ml of PM2.5 solution for 48h. After treatments, total RNA was isolated from cultured cells using Trizol reagent (Takara, Japan) and quantified using a Nano-Drop-1000 spectrophotometer (Thermo Fisher Scientific, USA). Reverse transcription was carried out using primeScript® RT reagent Kit (BIO-RAD, USA). RT-qPCR reactions were performed using SYBR Green Master-Mix (Applied Biosystems, USA) with 2 μl of template cDNA and 10 pmol of each primer on ABI 7300 system (Applied Biosystems, USA) according to the manufacturer’s instructions. Relative expression of mRNA to U6 or GAPDH was calculated using the 2^−ΔΔCt^ method to evaluate gene expression. The sequences of the primers were: miR-16-1-3p, Forward: 5’-GGGGCCAG-TATTAACTGT-3’, Reverse: 5’-TGCGTGTCGTGGAGTC-3’; U6, Forward: 5’-GCTTCGGCAGCACATATACTAAAAT-3’, Reverse: 5’-CGCTTCACGAATTTGCGTGTCAT-3’; Twist1, Forward: 5’-AAGCTGCAGCTATGTGGCTCACG-3’, Reverse: 5’-AATCACTGTCCACGGGCCTGTCT-3’; GAPDH, Forward: 5’-AGAAGGCTGGGGCTCATTTG-3’, Reverse: 5’-AGGGGC-CATCCACAGTCTTC-3’; α-SMA, Forward: 5’-ACCCAGAT-TATGTTTGAGACC-3’, Reverse: 5’-GCAGTTCGTAG-3’; E-cadherin, Forward: 5’- AAAGGCCCATTTCCTAAAAACCT-3’, Reverse: 5’- TGCGTTCTCTATCCAGAGGCT-3’; Vimentin, Forward: 5’-ACCGCTTCGCCAACTACAT-3’, Reverse: 5’-CTCCTGGAT’IffCCTCATCG-3’.

### 2.6 Scratch would healing assay

SMMC-7721 cells were seeded into six-well plates. When reaching 90% confluence, cells were treated with PM2.5. The scratches were created by drawing two parallel lines with a 10 μl pipette tips, and the floating cells were removed by gentle washing with PBS. Images were taken at 24h after scratches under a light microscope and the rate of cell migration was quantified.

### 2.7 Transwell invasion assay

Transwell filters (8μm pores) were inserted into a 24-well plate. The upper chambers were coated with 100 μl of diluted Matrigel (BD, USA) in serum-free RPMI-1640 medium and exposed to UV light for 2 h. A total of 3×104 cells were added to the upper chamber in serum free media, while RPMI-1640 medium containing 10% FBS was added to the bottom chamber. After 24 h incubation, the cells that migrated were fixed, stained with crystal violet, and observed under a microscope (Olympus Corporation, Japan) at 200× magnification. Five random fields in each replicate were chosen and counted. Results are presented as a ratio of cells that migrated relative to the cells that invaded in control group. Results are from six independent experiments.

### 2.8 Dual luciferase activity assay

3’UTR region sequence of Twist1 containing predicted miR-16-1-3p specific binding site was amplified by PCR from genomic DNA, and then inserted into the pGL3 luciferase reporter vector (Promega, USA) to obtain the wild-type luciferase reporter gene vector pGL-3-Twist1-wt. Several nucleotides were mutated in the predicted binding region of miR-16-1-3p, and this fragment was also cloned into pGL3 reporter vector to generate a mutant reporter plasmid pGL-3-Twist1-mut. All the constructed plasmids were verified through DNA sequencing. Constructed lucif-erase reporter plasmid pGL-3-Twist1-wt or mut and miR-16-1-3p or NC mimic were transfected into 293T cells using Lipofectamine 2000 reagent. After 24h, the cells were lysed and their luciferase activity was measured using a dual-luciferase detection kit according to the manufacturer’s instructions.

### 2.9 Statistical analysis

Data are presented as the mean ± the standard deviation (SD) from at least three independent experiments. All results were analyzed using the GraphPad Prism 5 software (GraphPad Software, San Diego, CA, USA). significance was analyzed using unpaired student’s t-test. *p*-values < 0.05 were considered statistically significant.

## 3 Results

### 3.1 Pro-proliferative effect of PM2.5 on SMMC-7721 cells

We first investigated the effect of PM2.5 on the growth of SMMC-7721 cells in vitro by CCK-8 assay. As shown in Figure 1A, exposing SMMC-7721 cells to PM2.5 for 24 h induced a dose-dependent increase in cell proliferation compared with the untreated cells. PM2.5 at a concentration of 25 μg/ml and 50 μg/ml caused a 30% (P) and 50% (P) growth enhancement in SMMC-7721 cells, respectively. We also examined the time-response relationship of PM2.5 (25 μg/ml) on SMMC-7721 cells. Incubating SMMC-7721 cells with media containing PM2.5 for 24 and 48 h had significantly promotion in cell growth (*p*<0.01) and similar effect with no significance (*p*>0.05) for 12h compared with the untreated cells (Fig. 1B).

**Figure 1:** Effect of PM2.5 on the growth of human SMMC-7721 cells (A) SMMC-7721 cells were cultured in the presence of various concentrations (5, 25, 50μg/ml) of PM2.5 for 24 h. Cell proliferation was measured by CCK8 assay. The optical density was then measured at 450 nm and the results were presented as percentage of control (arbitrarily set at 100%). All data shown are the of three separate experiments. (B) SMMC-7721 cells were cultured in the presence of 25 μg/ml PM2.5 for different time (12, 24, 48h). Cell proliferation was measured by CCK8 assay. The data were shown as the optical density measured at 450 nm. All data shown are the of three separate experiments. *, p < 0.05, **, p < 0.01.

### 3.2 Pro-metastatic potential of PM2.5 on SMMC-7721 cells

In order to evaluate the effect of PM2.5 on SMMC-7721 cell migration, an in vitro scratch wound assay was used. Scratch area was created both in PM2.5 treated and untreated wells, and the effect of PM2.5 on migration of SMMC-7721 cells was observed over a period of 24 h. As shown in Figure 2A, PM2.5 treated cells showed increased cell migration. To further investigate the invasive potential of PM2.5 treated cells, a transwell system coated with Matrigel was used. SMMC-7721 cells were seeded in the upper chamber and the percentage of migratory cells through the matrigel basement membrane after 24 h was quantified. Results (Fig. 2B) showed that PM2.5 treatment could increase the number of invaded cells compared with the untreated cells. Taken together, our data suggested that PM2.5 could markedly promote the ability of SMMC-7721 cells to migrate and invade in vitro.

**Figure 2:** Effect of PM2.5 on metastasis of human SMMC-7721 cells in vitro (A) Scratch wound assay was used to assess the effect of PM2.5 on SMMC-7721 migration at 24 h after PM2.5 treatment. Photographs were taken at 24h after scratch injury under ×200 original magnification. (B) Invasion ability of the cells were examined by transwell assay.

### 3.3 PM2.5 induced EMT in human SMMC-7721 cell lines

Since PM2.5 exposure has been demonstrated to induce epithelial mesenchymal transition (EMT) in tumor progression, it’s conceivable that PM2.5 might also trigger EMT in SMMC-7721 cells. We performed Western blot and RT-qPCR assays (Fig. 3) to analyze the expression of protein markers associated with EMT. Consistent with the observed morphological changes,The expressions of mesenchymal markers, vimentin and ɑ-smooth muscle actin (ɑ-SMA) were significantly increased, while the expression of epithelial marker, E-cadherin was found to be reduced markedly at both mRNA (Fig.3 A-C) and protein levels (Fig.3 A-D).

**Figure 3:** Potential of PM2.5 exposure on EMT in SMMC-7721 cells RT-qPCR was performed on (A) E-cadherin (B) Vimentin (C) ɑ-SMA expressions in PM2.5 treated SMMC-7721 cells in comparison to untreated cells. Results were normalized with the level of GAPDH control. (D) The expression levels of EMT related proteins were analyzed using Western blotting assay. GAPDH was used as the loading control. Data are presented as means ± SD. of three independent experiments. *, p < 0.05, **, p < 0.01.

### 3.4 miR-16-1-3p directly targets Twist1

Twist1 was predicted as a candidate target gene of miR-16-1-3p by bioinformatics (Fig.4A). To confirm the direct interaction between miR-16-1-3p and Twist1, a luciferase reporter construct containing a putative miR-16-1-3p-binding site of Twist1 3′UTR was generated as pGL-3-TWSIT1-wt, and mutant nucleotides were introduced into the predicted binding sequence to obtain pGL-3-TWSIT1-

**Figure 4:** miR-16-1-3p directly targets Twist1 (A) Sequence alignment shows the relative position of the miR-16-1-3p binding site in the 3′ UTR of Twist1 and the mutated nucleotides are indicated. The sequences were used to construct luciferase reporter plasmids. (B) SMMC-7721 cells were transfected with plasmids pGL-3-Twist1-wt or mut, along with miR-16-1-3p mimic or control. Dual luciferase assay was assayed at 24 h later. Luciferase activity was normalized to Renilla and presented as relative to miR control (arbitrarily set at 1). Data are presented as means ± SD. of three independent experiments. *, p < 0.05, **, p < 0.01.

mut (Fig. 4A). A dual luciferase reporter assay showed that miR-16-1-3p mimic was able to repress the luciferase activity of pGL-3-Twist1-wt, whereas pGL-3-Twist1-mut prevented this inhibition. These findings provided evidence that miR-16-1-3p could specifically bind to the predicted 3′UTR of Twist1.

### 3.5 Effect of PM2.5 on the expression of miR-16-1-3p level and its target Twist1

Since miR-16-1-3p is founded to be associated with the suppression of EMT in many cancers [29], the level of miR-16-1-3p mediated by PM2.5 was analyzed by RT-qPCR. SMMC-7721 cells were treated with PM2.5 for 24h and a significant repression of miR-16-1-3p was observed in PM2.5 treated SMMC-7721 cells (Fig.5A, p<0.01). Twist1, an important EMT transcription factor known to suppress E-cadherin transcription, was identified as a candidate target gene of miR-16-1-3p. Thus, we performed RT-qPCR and Western blotting assays (Figs. 5B and C) to examine the expression of Twist1 in PM2.5 treated SMMC-7721 cells. Significant inductions of Twist1 at mRNA and protein levels were

**Figure 5:** Effect of PM2.5 on the expression of miR-16-1-3p and Twist1 in SMMC-7721 cells (A) Expression of miR-16-1-3p in PM2.5 treated cells and un-treated cells was detected using RT-qPCR. (B) Expression of Twist1 in PM2.5 treated cells and un-treated cells was detected using RT-qPCR. (C) Expression of Twist1 in PM2.5 treated cells and un-treated cells was detected using WB. Results were normalized with the level of U6 control. Data are mean ± SD. *, p < 0.05, **, p < 0.01.

observed. Our data indicated the PM2.5 could repressed the expression of miR-16-1-3p, which was inversely correlated to that of its target Twist1.

### 3.6 Inhibitory effect of miR-16-1-3p on PM2.5 induced metastasis in SMMC-7721 cells

miR-16-1-3p mimic was used to study the effect of regulation of miR-16-1-3p on migration and invasion of PM2.5 treated SMMC-7721 cells. First, RT-qPCR data showed a significant increase in miR-16-1-3p expression in transfected SMMC-7721 cells compared with the non-transfected control (Fig. 6, p<0.01). As measured in in vitro scratch wound assay, miR-16-1-3p upregulation resulted in significant decrease in migration (Fig. 7A). A significant decrease in cell invasion was also observed at 48h following transfection with miR-16-1-3p using an in vitro transwell matrigel invasion system (Fig. 7B). Our data indicated that miR-16-1-3p could markedly suppress the metastatic ability of PM2.5 induced SMMC-7721 cells.

**Figure 6:** Transfection efficiency of miR-16-1-3p mimic in SMMC-7721 cells. SMMC-7721 cells were transfected with miR-16-1-3p mimic or negative control. Expression of miR-16-1-3p was detected at 24h post-transfection using RT-qPCR. Results were normalized with the level of U6 control. Data are mean ± SD. **, p < 0.01.

**Figure 7:** Effect of of miR-16-1-3p on PM2.5 induced metastasis in SMMC-7721 cells (A) Scratch wound assay was used to assess the effect of miR-16 on SMMC-7721 migration at 24 h after PM2.5 treatment. Photographs were taken at 24h after scratch injury under ×200 original magnification. (B) Effect of miR-16-1-3p on invasion ability was measured using transwell assays in PM2.5 treated SMMC-7721 cells.

### 3.7 Inhibitory effect of miR-16-1-3p on PM2.5 induced EMT in SMMC-7721 cells

Having confirmed the anti-metastatic potential of miR-16-1-3p, we next elucidated the possible mechanisms of miR-16-1-3p. Twist1 was identified as the target gene of miR-16-1-3p. Results from RT-qPCR and Western blotting assays revealed that miR-16-1-3p significantly inhibited the expression level of Twist1 (Fig. 8A and 8B). Twist1 was able to regulate some important genes associated with EMT and cell metastasis in cancer progression. Expressions

**Figure 8:** Effect of of miR-16-1-3p on PM2.5 induced EMT in SMMC-7721 cells (A) RT-qPCR was performed on gene expressions related to EMT in PM2.5 treated SMMC-7721 cells. Results were normalized with the level of GAPDH control. (B) The expression levels of EMT related proteins were analyzed using Western blotting assay. GAPDH was used as the loading control. Data are presented as means ± SD. of three independent experiments. *, p < 0.05, **, p < 0.01.

of vimentin and ɑ-SMA (the mesenchymal markers) were reduced, and expression of E-cadherin (the epithelial marker) was found to be upregulated at mRNA and protein levels as measured by RT-qPCR and Western blotting assays (Fig. 8A and 8B).

## 4 Discussion

China is experiencing extremely serious air pollution, and PM2.5 has become one of the main pollutants with health concerns in China [2, 5]. Due to the features of small size, strong adsoption, and complex constitution, PM2.5 can carry heavy metals and sulfates, etc, into human respiratory tract and lungs to induce multiple diseases including cancers [17, 20]. Recent studies have illustrated an association between PM2.5 and the incidence and progression of liver cancer [15, 16], however, the effect of PM2.5 on HCC and its possible mechanisms remain to be illustrated.

The present study showed that PM2.5, at a concentration of 25 μg/ml, displayed pro-proliferative and pro-metastatic effects on SMMC-7721 HCC cell line, consistent with the recent study taken by Qian Zhang [20]. The growth and metastasis promotive effects of PM2.5 was appeared to be associated with the induction of EMT process. To validate EMT conversion induced by PM2.5, morphological changes and EMT related marker genes were analyzed. Data revealed that SMMC-7721 cells exposure to PM2.5 displayed a morphological transition from a epithelial phenotype to mesenchymal phenotype. Accompanied with this, tThe induction of the mesenchymal markers (vimentin and ɑ-SMA) and the suppression of the epithelial marker (E-cadherin) was obviously observed in SMMC-7721 cells treated with PM2.5.

miR-16 has been reported to suppress the proliferation, invasion, and metastasis of HCC cells by mediating EMT process [25]. Twist1, identified as the direct target of miR-16, is reportedly to be an important transcription factor for regulating EMT process. Up-regulation of Twist1 has led to an EMT morphological transition as well as enhanced cell metastasis by mediating the expression E-cadherin, N-cadherin, and metalloproteinase [27, 28, 29]. miR-16 has been demonstrated to inhibit cell invasion and metastasis via inversely regulating Twist1 in some cancers such as gastric cancer and non-small cell lung carcinoma (NSCLC) [25, 26].

In our study, we noted that PM2.5 exposure resulted in the down-regulation of miR-16 expression and up-regulation of Twist1, and miR-16 mimic could enhance the metastasis and EMT process of SMMC-7721 cells exposure to PM2.5 by inversely regulating Twist1 expression, which were similar with the previous studies. Furthermore, dual Luciferase reporter assay confirmed the specifically binding of miR-16 to the predicted 3′UTR of Twist1.

## 5 Conclusion

Taken together, our study confirmed the pro-proliferative and pro-metastatic effect of PM2.5 on HCC cell line SMMC-7721. The possible mechanisms were EMT process induced by PM2.5 in SMMC-7721 cells, which was accompanized by an decrease in miR-16 and increase in Twist1 expression. miR-16 mimic could inhibit EMT changes induced by PM2.5 mainly through the down-regulation of Twist1 expression. Our findings might represent a key mechanism involved in PM2.5 air pollution, in order to advance our understanding of its impact on human health and improve the curative effects.
